This article has been retracted.

# Designing an intelligent monitoring system for corn seeding by machine vision and Genetic Algorithm-optimized Back Propagation algorithm under precision positioning

**DOI:** 10.1371/journal.pone.0254544

**Published:** 2021-07-15

**Authors:** Jiangtao Ji, Yayuan Sang, Zhitao He, Xin Jin, Shengsheng Wang

**Affiliations:** College of Agricultural Equipment Engineering, Henan University of Science and Technology, Luoyang City, China; Ministry of Natural Resources North Sea Bureau, CHINA

## Abstract

**Objective:**

To realize the regulation of the position of corn seed planting in precision farming, an intelligent monitoring system is designed for corn seeding based on machine vision and the Genetic Algorithm-optimized Back Propagation (GABP) algorithm.

**Methods:**

Based on the research on precision positioning seeding technology, comprehensive application of sensors, Proportional Integral Derivative (PID) controllers, and other technologies, combined with modern optimization algorithms, the online dynamic calibration controls of line spacing and plant spacing are implemented. Based on the machine vision and GABP algorithm, a test platform for the seeding effect detection system is designed to provide a reference for further precision seeding operations. GA can obtain better initial network weights and thresholds and find the optimal individual through selection, crossover, and mutation operations; that is, the optimal initial weight of the Back Propagation (BP) neural network. Field experiments verify the seeding performance of the precision corn planter and the accuracy of the seeding monitoring system.

**Results:**

1. The deviation between the average value of the six precision positioning seeding experiments of corn under the random disturbance signal and the ideal value of the distance is less than or equal to 0.5 cm; the deviation between the average value of the six precision positioning seeding experiments of corn under the sine wave disturbance signal (1 Hz) is less than or equal to 0.4 cm; the qualified rate of grain distance reaches 100%. 2. The precision control index, replay index, and missed index of the designed corn precision seeding intelligent control system have all reached the national standard. During the operation of the seeder, an alarm of the seeder leaking occurred, and the buzzer sounded and the screen displayed 100 times each; therefore, the reliability of the alarm system is 100%.

**Conclusion:**

The intelligent corn seeder designed based on precision positioning seeding technology can reduce the seeding rate of the seeder and ensure the stability of the seed spacing effectively. Based on the machine vision and GABP algorithm, the seeding effect detection system can provide a reference for the further realization of precision seeding operations.

## 1. Introduction

Agriculture is not only the main industry of China but also one of its economic pillars. Due to factors such as climate change, population growth, and food security, the agricultural sector needs more innovative methods to increase its crop yields [1, 2]. In recent years, with the steady rise of artificial intelligence (AI) technologies, relevant applications have gradually penetrated the entire process of agricultural production. Among AI technologies, machine learning, computer vision, big data analysis, and cloud computing are the most widely used ones. As an important food crop and cash crop in China, corn is widely distributed and covers the main food-producing areas in China [3–5]. Therefore, research on corn planting is of great significance to the development of primary and secondary industries in China.

As China ‘s agricultural seeding methods have also entered a new stage of development, the current precision seeding technology, as a mechanized planting technology, not only reduces manual labor but also ensures accurate and consistent seeding volume, thereby making reasonable plantation allocation and increasing the yield of crops [6]. Precision seeding sows a determined number of seeds at a determined depth according to a determined row and grain spacing; meanwhile, it covers the seeds with an appropriate amount of wet soil and compact the soil using a moderate pressure and strength. Precision seeding undergoes two developmental stages, namely, quantitative hole seeding and single seed on-demand seeding. Quantitative hole seeding was first applied to crops such as corn and cotton. This method is beneficial to the field protection of seedlings when the plant protection and seed selection and processing techniques are not perfect. As of now, the seedling rate and seedling protection rate in the field can be well guaranteed with the development of science and technology, the gradual popularization of fine seeds and selection techniques, the widespread application of modern plant protection technology and irrigation technology. Hence, single-seed precision seeding has developed rapidly. However, the actual operation of precision seeders in China also has some problems, such as unstable seeding and untimely operation monitoring and alarm. Therefore, improving the work quality and efficiency of no-till seeders is of great significance to agricultural production stability and income increase [7]. The application of modern scientific and technological achievements in agriculture is a general trend in the development of agricultural technology.

At present, some large agricultural machinery companies worldwide already have quite advanced technologies in the field of no-tillage seeders, producing a variety of models and a series of intelligent sowing and fertilizing machines. The model 1006NT no-tillage seeder produced by Great Plains Mfg. Inc. (the USA) has sophisticated technology but a low price. It can complete multiple procedures such as trenching, fertilization, seeding, and earthing at one time, which achieves the precision seeding where one seed occupies one hole with the same seeding depth. Globally, most agricultural machinery companies have installed real-time monitoring systems on their no-tillage seeders. In China, companies and scientific research institutions have also done a lot of work in this regard. The model produced by Heilongjiang Agricultural Machinery Institute, 2BJM-6 no-tillage seeder, is a 6-row sowing seeder, which has a row spacing of 60–70 cm and is suitable for the sowing of corn, soybean and other crops [8]. The model is well-shaped and has good adaptability to the complex working environment of farmland. Also, it can achieve precision seeding. At present, a gap exists between China’s research on the precision sowing monitoring system and that of the US and Europe. Therefore, in-depth research is needed in the monitoring of sowing conditions and the stepless regulation of sowing distance. The on-line monitoring-based intelligent precision positioning and seeding with multiple information fusion will be the development direction of precision seeding technology in China [9]. Many factors are influencing agricultural mechanization, and the degree of influence is uncertain. In the past, methods to research agricultural mechanization are mostly linear regression econometric models, difficult to truly describe the complex nonlinear relationship between agricultural mechanization and the influencing factors.

To achieve the regulation of the seed position in precision seeding, this study conducts research on precision positioning seeding technology, comprehensively applies technologies such as sensors and Proportional Integral Derivative (PID) controllers, and combines modern optimization algorithms to implement online dynamic calibration control of line spacing and plant spacing. The system can reduce the seeding rate of the seeder to lay a foundation for improving the precision control of variable fertilization. At the same time, it provides a theoretical basis and technical reference for the development of precision positioning seeding technology and system devices. Therefore, based on the machine vision and Genetic Algorithm-optimized Back Propagation (GABP) algorithm, a test platform for the seeding effect detection system is designed to provide a reference for further precision seeding operations.

## 2. Experimental procedure

### 2.1 Design of intelligent control system for corn precision seeding

As an important element in the structure of the seeder, the quality of the seeder will directly affect the working performance of the seeder [10–12]. Fig 1 shows a structural diagram of a corn precision seeder designed in this study. The front simulation wheel of the seeder is used instead of the traditional tractor front wheel. The simulated wheel has a larger load-bearing; therefore, the slip rate is very low. This can make the ground wheel speed more stable and avoid the occurrence of missed planting. In addition, a monitoring device installed at the bottom of the seed metering device can monitor the drop of seeds; at the same time, it can monitor the non-seeding caused by the incomplete filling of the seed box.

**Fig 1:** General structure of a corn precision seeder.

During normal operation of the corn seeder, the fan rotates at high speed and generates a negative pressure in the vacuum chamber of the seeder. The corn seeds are adsorbed on the seeder tray and rotate with it; when the seeds are out of the vacuum chamber, they will drop into the seed tube due to their gravity [13]. During the operation of corn precision seeding, the controller collects the information of force sensor in real-time and compares it with the threshold value of the set force sensor, ensuring the pressure values of the depth-limiting wheel and the ground surface are within the set threshold range, thereby maintaining the stability of ditch depth. Therefore, the planting depth of corn is as consistent as possible.

Among the various parts of the seeder, the performance of the seeding device directly affects the seeding performance of the seeder. The finger-clip seeding device has the advantages of balanced seed discharge, low seed damage rate, and simple structure; therefore, it is widely used in agricultural production [14, 15]. When the seeding device works, the finger clip passes through the filling area, and the corn seeds are squeezed into the space between the finger clip and the seed plate. Then, the finger clip clamps the corn seeds and pushes the corn seeds to rotate into the seed cleaning area. The brush is used for seed cleaning so that the seeds fall on the seed guide belt behind the seeding device. The seeds rotate with the seed guide belt and eventually fall into the flexible seed tube under the effect of their gravity, which is guided by the flexible seed tube. Therefore, the precise, low-speed, and uniform seeding of corn seeds is achieved [16]. When the corn seeds are thrown away from the seed guide belt, in a plane parallel to the rotation of the seed meter, the corn seeds will generate an initial speed V_x_ in the horizontal direction opposite to the advance direction of the machine due to the rotation of the seed guide belt. At the same time, under the action of gravity, the seed will generate a vertical downward speed V_z_. Since the position of the corn on the seed guide blade and the centerline position of the conveyor belt have a certain deviation, there is also a centrifugal force component in the rotation plane perpendicular to the seeder. Therefore, the seed produces a horizontal initial speed perpendicular to the advance direction of the machine V_y_. Its speed model is shown in Fig 2.

**Fig 2:** Speed model of the seeding device.

Kinematics analysis of the corn seeds at the exit of the seed tube is performed. A rectangular coordinate system OXZ on the rotation plane of the seed guide belt is established, and the coordinate origin O coincides with the seeding point of the tube mouth. Then, a rectangular coordinate system PYZ is established, the coordinate origin that is perpendicular to the rotation plane P coincides with the center of the seed tube. The movement track of corn seeds is:

$$\left\{ \begin{array}{l} X=V_{X}t\\ Y=V_{Y}t\\ Z=V_{Z}+gt^{2}/2 \end{array}\right.$$ (1)

Where: X refers to the front horizontal displacement (mm), Y refers to the lateral horizontal displacement (mm), and Z refers to the vertical-horizontal displacement (mm); t is the movement time of the corn seeds (s), V_x_ refers to the frontal horizontal component (m/s) of the seeding speed, V_y_ refers to the lateral horizontal component (m/s) of the seeding speed, and V_z_ refers to the vertical component (m/s) of the seeding speed. When the rotation speed of the seeding shaft of the seeding device, the position of the seeding tube with respect to the seeding device, and the tilting angle of the seeding device are changed, the collision situation will also change, and the seeding situation of the seeds will change immediately.

In the practical application of the seeder, the PID controller is a widely used control method [17]. **In this study, the PID controller is used to realize the real-time matching between the working forward speed and the rotation speed of the finger-clip seeding device.** The PID controller can adjust the input value according to the historical data and the occurrence rate of the difference, which makes the system more accurate and stable. PID controller can achieve synchronous matching between the working speed of the machine tool and the speed of the finger-clamp-type seed metering device. Once other control methods cause system stability errors or process repetitions, the PID feedback loop can stabilize the system. The PID controller can be expressed as:

$$u(t)=K_{p}+K_{i}\int_{0}^{t}e(\tau )d\tau +K_{d}\frac{de(t)}{dt}$$ (2)

Where: *K*_*p*_, *K*_*i*_, and *K*_*d*_ respectively represent the proportional coefficient, the integral coefficient, and the differential coefficient of the PID controller. These three parameters directly determine the performance of the PID controller. The PID control system model built in Simulink is shown in Fig 3. From a signal transformation perspective, lead correction, lag correction, and lag-lead correction can be summarized as three operations, proportional, integral, and derivative, and their combinations. The application scope of PID regulator: PID is a traditional regulation control method, suitable for almost all sites such as temperature, pressure, flow, and liquid level. On different sites, only the PID parameters should be set differently; as long as the parameters are set properly, good results can be achieved.

**Fig 3:** Model of PID control system.

### 2.2 The intelligent monitoring system for corn precision seeding

Aiming at the self-detection needs of the seeder, this study designs a seeding effect detection system based on machine vision, conducts a seeding detection test, and improves the automation level of the machine.

(1) Hardware system: The corn seeding detection system uses a precision seeder as an experimental platform. The hardware of the seeding detection test platform mainly includes a power source, a computer, a camera, a light source, and a seedling tray. The parameters of the camera are shown in Table 1, the hardware system of corn precision seeding is shown in Fig 4.

**Fig 4:** Hardware system of corn precision seeding.

**Table 1:** Camera parameters of the inspection system.

Model	Mind Vision MV-GE200GC-T
Resolution	2 million pixels
Sensor type	CMOS
Exposure mode	Frame exposure
Pixel size	4.5 μm
Frame rate	60
Target size	1/1.8
Minimum exposure time	0.015 ms
Color	Multicolor
Collection mode	Continuous, software triggered, hardware triggered

The seedling tray is gray, and the corn seeds are yellow-brown. Considering that the imaging effect when shooting the seedling tray is affected by the light intensity and light source color on the seed target, while the yellow LED light source is advantageous for the reflection of the seed but disadvantageous for the seedling tray, the white LED light source that is advantageous for target reflection is selected. The light source in this study uses three LED strip light sources with a weight of 5 wt, and the top side is illuminated in the form of scattered light. According to the height between the camera plane and the seedling tray, the lens with a suitable focal length is selected.

(2) Software system: The software system for monitoring the specific situation of corn seeding mainly includes three sections: collection, processing, and display. The function library of LabVIEW includes data acquisition, GPIB, serial port control, data analysis, data display, and data storage. Matlab is a high-level matrix language that includes control statements, functions, data structures, input and output, and object-oriented programming. This study is based on the powerful data acquisition capabilities of LabVIEW and the high computational efficiency of MATLAB. The LabVIEW program is selected for image acquisition and display, and MATLAB is selected for image processing. All images during acquisition, processing, and display are stored in the same folder. By using a sequential logical structure, three parts of the program are executed in sequence. The final imaging results are automatically displayed on the page. The specific values of the seeding qualification rate, replay rate, and missed rate are calculated.

### 2.3 Seed number recognition based on GABP

GA is a kind of bio-intelligence algorithm. It uses cross-variation of chromosomes of good individuals and retains the characteristics of good individuals to solve the problem [7, 18, 19]. In deep learning, no matter how complicated the structure is, it is necessary to solve the problem through three structures, i.e., model, strategy, and algorithm. The BP neural network in the field of deep learning is simple and practical, with high convergence speed and execution efficiency; however, the stability of the algorithm is poor [11]. Based on the analysis of the GABP algorithm, the GA is used to optimize the back-propagation neural network for weights and thresholds. The corresponding weights and thresholds are obtained so that the structure of the BP neural network can be controlled steadily and the problem can be solved quickly and efficiently, which improves the stability of the algorithm [2, 20, 21].

The topology of the three-layered neural network is shown in Fig 5. The input layer of the BP network has n nodes, the hidden layer has q nodes, and the output layer has m nodes. Therefore, the BP network has completed the approximate mapping of n-dimensional space vectors to m-dimensional space. When the number of pattern samples is large, it is necessary to reduce the network scale and add a hidden layer. However, the number of hidden layers of a BP network generally does not exceed two.

**Fig 5:** Topology of a three-layered neural network.

The GABP algorithm can better predict the output of the function. First, the connection weight of the input layer and the hidden layer, the hidden layer threshold, the connection weight of the hidden layer and the output layer are encoded. The individual fitness value (F) can be expressed as:

$$F=k(\sum_{i=1}^{n}abs(y_{i}-o_{i}))$$ (3)

Where: *y*_*i*_ indicates the expected output of the i-th node, *o*_*i*_ indicates the predicted output of the i-th node, and k is the coefficient.

The selection probability of the individual i of the selection operation can be expressed as:

$$p_{i}=f_{i}/\sum_{i=1}^{N}f_{i}$$ (4)

$$f_{i}=k/F_{i}$$ (5)

Where: *F*_*i*_ is the fitness value of individual i, N is the number of individuals in the population, and k is the coefficient.

In the cross operation, the real number cross method is used. The k-th and l-th chromosomes are denoted as *a*_*kj*_ and *a*_*lj*_, respectively, and the cross operation method is expressed as:

$$a_{kj}=a_{kj}(1-b)+a_{lj}b$$ (6)

$$a_{lj}=a_{lj}(1-b)+a_{kj}b$$ (7)

In the mutation operation, the j-th gene *a*_*ij*_ of the i-th individual is selected for mutation, and the operation method is expressed as:

$$a_{ij}=\{\begin{array}{l} a_{ij}+(a_{ij}-a_{\min})\times f(g),r\leq 0.5\\ a_{ij}+(a_{ij}-a_{\max})\times f(g),r>0.5 \end{array}$$ (8)

$$f(g)=r_{2}{\left(1-g/G_{\max}\right)}^{2}$$ (9)

Where: r is a random number, g is the current number of iterations, *G*_max_ is the maximum number of evolutions, and *a*_min_ and *a*_max_ are the upper and lower bounds of *a*_*ij*_, respectively.

Generally, the weights and thresholds of the neural networks are stochastically initialized to random numbers between [–1, 1]. This initialized parameter has a great influence on the training of the network. The global optimization feature of GA is used to search for the random solution that can replace the initial value. Then, the local search feature of the BP algorithm is utilized to find the optimal solution. After one network training and one prediction, the norm of the test error is used as the right GA to calculate the fitness value. After calculation, the optimal weights and thresholds are obtained and assigned to the new neural network. when the maximum genetic algebra or training error is reached or the requirements are met, the overall cycle ends. After the structure of the BP neural network is determined, the GABP network training is performed. Fig 6 shows the training flow of the GABP algorithm. Based on the global optimization feature of GA, a random solution that can replace the initial value is searched. To obtain the optimal solution, it is necessary to continue to apply the BP algorithm for local search.

**Fig 6:** Training flow of GABP algorithm.

GABP introduces GA into the training process of BP neural network and uses network weights and thresholds as population individuals to imitate genetic codes. It uses the sum of the absolute value of the sample predicted value and the observed value of the error as the individual fitness function. The optimal individual in the population can be finally obtained through continuous iterative evolution operations, including selection, crossover, and mutation. After decoding, the global optimal weights and thresholds of BP neural network are obtained. Thus, BP neural network optimized by the genetic algorithm is established. In summary, the purpose of the GABP algorithm is to obtain better initial network weights and thresholds through genetic algorithms. The basic idea is to use the initial weights and thresholds of individual representative networks and the BP neural network initialized by individual values. The prediction error is used as the fitness value of the individual, and the optimal individual is found through selection, crossover, and mutation operations, i.e., the optimal initial weight of the BP neural network.

The general detection flow is shown in Fig 7. From left to right and from top to bottom, each seedling hole is sequentially inspected first; then, the connected domain in each seedling hole is detected. In the training process, the actual output of each connected domain is a matrix with 1 row and 2 columns. To represent the number of seeds contained in each connected domain with numbers, the matrix is reduced in dimension. It is assumed that the output of the i-th connected domain in each seedling hole is (m, n), where *a*_*i*,1_ = *m* and *a*_*i*,2_ = *n*; then, the output after dimension reduction is: *a*_*i*,3_ = 2^0^×*a*_*i*,1_+2^1^×*a*_*i*,2_. If the output result is 0, the hole is empty; if the output is in the range of (0, 1), there will be 1 super seed; if the output is in the range of (1, 2), there will be 2 super seeds; if the output is in the range of (2, 3), there will be 3 super seeds. The algorithm is divided into two parts for implementation. According to the theoretical basis, GA is utilized to improve the BP neural network (BPNN), find the optimal weights and thresholds, and create and train the network model. The overall detection method is determined. Afterward, each seedling hole is detected successively from left to right and from top to bottom. Then, the connected domain in each seedling hole is detected, and the shape characteristic parameters of the connected domain are extracted to form a test set. The test set is loaded, and the number of super seeds represented by all connected fields in a single seedling hole is accumulated as the final output result and displayed in the matrix of LABVIEW.

**Fig 7:** The overall process of visual inspection based on GABP algorithm.

### 2.4 Field experiments of corn seeding

To verify the accuracy of the intelligent seeding monitoring system, this study will verify the seeding performance of the precision seeder through field experiments. The corn seed variety used in this experiment was Denghai 6702, with a water content of 14.7%, a medium constant of 1.8, and a horse-tooth shape appearance. Other equipment required for experiments include tractors, tape measure, and notebooks.

The field trial was conducted in July 2019 in the experimental field of Henan University of Science and Technology Agricultural Production Materials Co., Ltd. in Henan Province, China. The number of operation rows was two, and three measurement areas with a length of 10 m were randomly selected. A total of 6 corn reseeding experiments were performed. The soil covering device of the seeder can be removed to facilitate the measurement work. Before seeding, the tractor speed should be stabilized before passing through the test area at a uniform speed. During the seeding process, the operating speed of the tractor should be maintained at 5–8 km/h. After the seeder passes, the seed distance in the test field is measured with a tape measure. The method for measuring the seed distance is to measure the projection distance of the center of two adjacent seeds on the seeding centerline, and the measurement unit is cm.

## 3. Results and discussion

### 3.1 Test results of stability of corn seed distance

Generally, the distance between spring seeding corn plants is 33–40 cm, and the distance between summer seeding corn plants is 25–33 cm. Therefore, in this test, the corn seed distance was set to be 30 cm, and the corn seed stability test was completed under this condition. According to agronomic parameters, the running speed of the conveyor belt is set to 1.5 m/s, the seeding interval between two seeds is 0.2 s, 8 seed holes are set on the mechanical seeding plate, and the rotation speed of the seeding plate is 30 r/min. A total of 6 repeated corn seeding experiments were performed, and the results of the precision seeding experiments of the corn under the random perturbation signal and the sine wave perturbation signal (1 Hz) were shown in Figs 8 and 9, respectively.

**Fig 8:** Precision positioning seeding experiment of corn under random disturbance signals.

**Fig 9:** Precision positioning seeding experiment of corn under sine wave disturbance signal (1 Hz).

Under the random disturbance signal, the average grain distances of the 6 corn precise positioning seeding experiments were 29.5 cm, 29.3 cm, 29.7 cm, 30.2 cm, 29.8 cm, and 30.4 cm, respectively. The deviation from the ideal grain distance of 30 cm was less than or equal to 0.5 cm. The average grain distances of the 6 precise corn seeding experiments under a sine wave disturbance signal (1 Hz) were 29.6 cm, 30.0 cm, 30.0 cm, 29.8 cm, 30.2 cm, and 29.7 cm, respectively. The deviation from the ideal grain distance of 30 cm was less than or equal to 0.4 cm. The measured values of the grain distance of the 6 precise corn seeding experiments under the random disturbance signal and the sine wave disturbance signal (1 Hz) were in the range of 24 cm to 36 cm, i.e., the grain spacing qualified rate reached 100%.

Traditional BP neural network revises the network weights and thresholds using gradient descent. It is easy to fall into local extreme values and cannot find the global optimal solution. GA can search for the global optimal solution randomly by simulating the natural evolution process. GABP introduces GA into the training process of BP neural network and uses network weights and thresholds as population individuals to imitate genetic codes. It uses the sum of the absolute value of the sample predicted value and the observed value of the error as the individual fitness function. The optimal individual in the population can be finally obtained through continuous iterative evolution operations, including selection, crossover, and mutation. After decoding, the global optimal weights and thresholds of BP neural network are obtained. Thus, BP neural network optimized by the genetic algorithm is established.

### 3.2 Overall situation of corn seeding and results of system tests

According to the performance specifications of precision seeders regulated in *JBT 10293–2013 Single-Grain (Precision) Seeder Technical Conditions* [22], when the distance between the seeding plant X≥ 20 cm, if the qualified index of plant distance≥ 80%, the re-seeding index≤ 5%, the missed index≤ 8%, the precision performance of the precision seeder has reached the standard. By calculating the index of the single-grain operation test, the data obtained are shown in Table 2 and Fig 10.

**Fig 10:** Results of single-grain operation test indicators.

**Table 2:** Calculation results of single-grain operation test indicators.

Test serial number	Plant spacing qualification index (%)	Replay seeding index (%)	Miss seeding index (%)
1	97.5	1.3	0.8
2	93.3	2.1	1.5
3	96.8	3.5	2.4
4	97.3	0.9	1.3
5	96.5	4.2	3.4
6	94.5	5.3	4.6

As shown in the data in Table 2, through 6 experiments, the plant precision index, re-seeding index, and missed index of the corn precision seeding intelligent control system designed in this study have reached the national standard. This shows that the control system designed in this study can effectively improve the uniformity of the seeder so that the operating quality and performance of the seeder can be ensured. During the operation of the seeder, an alarm of the seeder leaking occurred, and the buzzer sounded and the screen displayed 100 times each. Therefore, the reliability of the seeder missed alarm and the overall alarm system is 100%.

## 4. Conclusion

Precision positioning corn seeding refers to the seeding technology that uses precisely positioned corn seeding machines to place corn seeds in the soil in a fixed amount according to the precise row spacing, plant spacing, and seeding depth according to the requirements of modern agronomy. At the same time, the precision positioning of corn seeding can make the cornfield neat and tidy. Also, combined with the corn breeding technology, it is beneficial to the later mechanized corn harvesting. In this study, through research on precision positioning seeding technology, and implementing online dynamic calibration control of line spacing and plant spacing, the results provide a theoretical basis for the development of precision positioning seeding technology and system devices.

When designing the control system of the seeder in this study, the effective series seeder and flexible seed tube work together to complete the seeding and guiding functions. A monitoring device is installed at the bottom of the seeding device, which can monitor the drop of seeds; at the same time, it can monitor the non-seeding caused by the incomplete filling of the seed box. In this study, the PID controller is used to realize the real-time matching between the working forward speed and the rotation speed of the finger-clip seeding device. The PID controller can adjust the input value according to the historical data and the occurrence rate of the difference, which makes the system more accurate and stable. To verify the accuracy of the intelligent seeding monitoring system, this study verifies the seeding performance of the precision seeder through field experiments based on the seeding detection method of the GABP algorithm. A total of 6 repeated corn seeding experiments were carried out. According to the results of the precision positioning of the seed distance of the corn under a random disturbance signal and a sine wave disturbance signal (1 Hz), it was found that the grain spacing qualified rate reached 100%. During the operation of the seeder, an alarm of the seeder leaking occurred, and the buzzer sounded and the screen displayed 100 times each. the reliability of the seeder missed alarm and the overall alarm system is 100%.

The intelligent corn seeder designed based on precision positioning seeding technology can reduce the seeding rate of the seeder and ensure the stability of the seed spacing effectively. Based on the machine vision and GABP algorithm, the seeding effect detection system can provide a reference for the further realization of precision seeding operations. Due to the limitation of time, only the preliminary research on the seed distance is conducted in this study. In the subsequent research, the depth of the seed needs to be discussed to fully evaluate the performance of the intelligent seeder.

## Supporting information

S1 Data (XLSX)
